The article "Application of Genetic Algorithm and U-Net in Brain Tumor Segmentation and Classification: A Deep Learning Approach" was published in 2022. Journal: Comput Intell Neurosci.

# Application of Genetic Algorithm and U-Net in Brain Tumor Segmentation and Classification: A Deep Learning Approach

**DOI:** 10.1155/2022/5625757

**Published:** 2022-09-15

**Authors:** Muhammad Arif, Anupama Jims, Ajesh F., Oana Geman, Maria-Daniela Craciun, Florin Leuciuc

**Affiliations:** ^1^Department of Computer Science, Superior University, Lahore, Pakistan; ^2^Department of Computer Science and Information Technology JAIN (Deemed-to-be University), Bangalore, India; ^3^Department of Computer Science and Engineering, Sree Buddha College of Engineering, Pattoor Alappuzha, Kerala, India; ^4^Stefan Cel Mare University of Suceava Romania, Suceava, Romania

## Abstract

The development of unusual cells in the cerebrum causes brain cancer. It is classified primarily into two classes: a noncarcinogenic (benign) type of growth and cancerous (malignant) growth. Early detection of this disease is a quintessential task for all medical practice professionals. For traditional approaches of tumor detections, certain limitations exist. They include less effectiveness, inability to detect due to low-quality processing of images, less dataset for training and testing, less predictive nature to models, and skipping of quintessential stages. All these lead to inaccurate results of tumor detections. To overcome this issue, this paper brings an effective deep learning technique for brain tumor detection with the following stages: (a) data collection from REMBRANDT dataset containing multisequence MRI of 130 patients; (b) preprocessing using conversion to greyscale, skull stripping, and histogram equalization; (c) segmentation uses genetic algorithm; (d) feature extraction using discrete wavelet transform (DWT); (e) particle swarm optimization technique for feature selection; (f) classification using U-Net. Experiment evaluation states that the proposed model (GA-UNET) outperforms (accuracy: 0.97, sensitivity: 0.98, specificity: 0.98) compared to other advanced models.

## 1. Introduction

The brain is a vital part of the neurological system. The human brain and nerve system are linked by the bone marrow. Our brain is the primary controller of all human behaviors and activities. It takes data from all of the sense organs, makes a choice, and transmits instructions to the relevant organ. The brain, with the aid of neurons, manages all of the actions of the human body.

The two most common forms of brain tumors are malignant and benign. It is believed to be the most lethal malignancy in both adults and children alike. When tissues multiply abnormally, a tumor forms. The creation of a mass of cells that subsequently changes into tumors is caused by abnormal tissue growth relative to normal healthy cells [1]. Cancer is caused by the proliferation of cancerous tumor cells. The malignant tumor cells have spread throughout the brain. Pituitary glioma and meningioma are the most frequent tumors identified in adults. Gliomas are tumors that develop from glial cells found in the brain's secondary tissue. Various glands like the thyroid are controlled by hormones produced from the pituitary. The functioning of these glands will be disrupted by a pituitary tumor (National Brain Tumor Society).

It is critical to identify the tumor as soon as possible in order to cure it. The accuracy rate of tumor detection is mostly determined by the procedures employed for tumor detection and the experience and professional abilities of the doctors involved. Finding the proper sort of brain tumor early on might be difficult, but it is crucial since it allows doctors to treat the patient appropriately [2]. Medical image processing is critical in assisting humans in the diagnosis of many disorders. Computer tomography (CT) and magnetic resonance imaging (MRI) are the two methods utilized to identify the tumor in its early stages. These two approaches can be used to detect anomalies in brain tissues, such as cell size, position, or form [3].

Strong deep learning systems improve the accuracy of the identification and thus support clinicians in planning further treatment processes. An efficient algorithm with appropriate properties and classifiers must be chosen to achieve optimum efficiency. In comparison with the previous manual categorization method, algorithms are more efficient and exact [4].

### 1.1. Key Highlights

This paper brings an operative deep learning layout for brain tumor detection. The following are the key highlights:

- An efficient deep learning style for brain tumor detection and classification
- Segmentation is done using a genetic algorithm for segmenting the tumor regions
- Feature extracted and selected using PCA and PSO
- Sorting of brain tumor imaginings using U-Net network
- Evaluation results bring the effectiveness of the proposed models

Organization of paper: since we previously covered the overview of brain tumors and their deep learning viewpoint in Section 1, the rest of the research is organized as follows.  Section 2 is a review of the literature, Section 3 is the representation of the updated approach, Section 4 is the representation of the performance measures, and Section 5 is the conclusion.

## 2. State-of-the-Art Models

Khan et al. [5] breaks down the process into five main parts. To begin with, edge-based histogram equalization and the discrete cosine transform (DCT) were used to create the linear contrast stretching. The next step is to extract deep learning characteristics. Transfer learning was used to extract features from two pretrained convolutional neural network (CNN) models, VGG16 and VGG19. In the third step, the extreme learning machine was employed in conjunction with a correntropy-based joint learning technique to find the best characteristics (ELM). The produced matrix is then sent to ELM for further categorizing. The suggested method was validated using the BraTS datasets, yielding accuracy rates of 97.8%, 96.9%, and 92.5% for BraTs2015, BraTs2017, and BraTs2018, respectively.

Sangeetha et al. [6] provided a classifier with several iterations based on many CNN architectures. For the next 60 iterations, VGGNet has an accuracy rate of 89.33%, Google Net has a rate of 93.45%, and ResNet 50 has a rate of 96.50%. Finally, it is demonstrated that ResNet 50 outperforms VGG Net and GoogleNet in terms of speed and accuracy.

Naser and Deen [7] created a CNN-capable UNet. The segmentation and grading algorithms were trained and validated using T1-precontrast, FLAIR, and T1-postcontrast MRI data from 110 patients with lower-grade glioma (LGG). The mean Dice similarity coefficient (DSC) and tumor detection accuracy of the segmentation model are 0.85 and 0.93, respectively.

Saleh et al. [8] proposed to use AI Algorithms, CNN, and deep learning to improve the quality and efficiency of MRI scanners in categorizing brain tumors and identifying their kinds. We used five pretrained models to train our brain tumor dataset: Xception, ResNet50, InceptionV3, VGG16, and MobileNet. For unseen images, the *F*1 scores were 98.75%, 98.50%, 98.00%, 97.50%, and 97.25%, respectively. These precisions help to discover malignancies early before they develop physical adverse effects like paralysis and other problems [9–14].

## 3. Methodology

Figure 1 shows the overall block of the proposed system for detecting brain tumors, with the following stages: (a) REMBRANDT data were collected for deep learning models. A total of 130 patients' multisequenced MRI pictures were gathered. These images contain sounds and irregularities that could interfere with the detection of brain tumors at later stages. As a result, (b) preprocessing is required to remove noise and abnormalities from raw photos. Greyscale conversion, skull stripping, and finally histogram evaluation were the three procedures utilized for this goal. The preprocessed images were then utilized to perform (c) segmentation, which involves using a genetic algorithm (GA) to segment tumor regions from the images. Then, from the segmented picture, specific features were extracted for (d) feature extraction using the discrete wavelet transform (DWT), followed by dimensionality reduction using (e) feature selection, which used PSO to optimize the features, and finally, classification. Brain tumors are classified using the U-Net approach.

### 3.1. Data Collection

This study made use of brain tumor datasets from the Repository of Molecular Brain Neoplasia Data (REMBRANDT) [15]. The REMBRANDT database comprises 110,020 presurgical MR multisequence images from 130 brain tumor patients. Among the tumors in the collection are astrocytes (AST), oligodendrogliomas (OLI), glioblastoma multiforme (GBM), and other unidentified tumors. The photos were all digitized at 256*∗*256-pixel resolution. Each picture in the REMBRANDT databases was linked to a certain type of brain tumor.  Figure 2 shows some REMBRANDT picture samples [16, 17].

### 3.2. Preprocessing

As images are collected, these are in raw format. So, chances of noise and anomalies may be large. So, to avoid this, preprocessing techniques are used. To preprocess the input MRI image, the RGB to grey conversion, skull strip removal, and histogram equalization techniques is employed.

#### 3.2.1. Grey Scale Conversion

After scanning, an image is created in the RGB (red, green, and blue) colour format. The image's three separate planes are made up of red, green, and blue components. In RGB pictures, pixel intensity is represented by a combination of these three plane intensity values. In a greyscale image, the intensity values represent pixel values that range from 0 to 256. Greyscale photos with various shades of grey ranging from black to white were used. The light intensity for each pixel in a greyscale picture is confined inside a single band of the electromagnetic spectrum [18, 19]. Converting a colour image to greyscale is done by altering the weighting of the colour channels red, green, and blue [4] accurately. The match between the brightness of the greyscale picture and the brightness of the RGB image determines the resemblance between the two images. To boost the brightness of the image, subtract 31% of the red value, 57% of the green value, and 15% of the blue value from the RGB image.  Figure 3 depicts both the original RGB image and the greyscale conversion.

#### 3.2.2. Skull Strip

Skull stripping is the removal of nonbrain anatomy and unwanted components from scanned images. Using the cerebrospinal fluid rim to eliminate the undesired pieces (CSF) was done. Using intensity thresholding, the skull may be removed, followed by a morphological technique to give the requisite brain area for tumor diagnosis. Allow the input picture to be represented as an array of pixels with intensity values at key points in the image [20].

(1) $$\begin{array}{c} Let\;Ip=\left\{Ip1,Ip2\ldots \ldots \ldots \ldots \ldots \ldots \ldots \ldots \ldots \ldots \ldots ,Ipn\right\}\text{.} \end{array}$$

The intensity values of pixels 1 to *n* are represented by *Ip*1…. *Ipn*. *pn* represents the total number of pixels in a picture. Let us suppose the intensity threshold is *T*, and the pixel intensity must be less than *T* to be removed from the image. Pixels that match this requirement would normally indicate thin connections. The intensity thresholding mask should also protect as much of the brain as feasible. In this case, selecting the appropriate threshold value is critical since setting it too low may result in the inclusion of unwanted garbage. High threshold values can help distinguish between the brain and nonbrain structures, but they come at the cost of brain degeneration. As a result, in order to achieve acceptable results, the threshold should be set at a suitable level.  Figure 4 shows a skull strip image taken from an MRI scan.

We now have the necessary brain imaging, which must be refined before it can be used for tumor detection. We employ morphological operations to accomplish this. It also aids in the elimination of tight connections.

#### 3.2.3. Histogram Equalization

To improve their quality, the acquired brain MR images need preprocessing. This allows for more accurate feature extraction. In this study, a method known as CLAHE was used. The majority of the photos in the datasets studied are of low contrast. CLAHE, an adaptive histogram equalization (AHE) version, calculates the intensity histogram in each pixel-centered contextual zone. The local histogram's pixel intensity is then converted to a value based on the pixel intensity level within the display range [21]. CLAHE, in contrast to AHE, limits contrast enhancement to reduce overenhancing of noise and edge shadowing [22]. CLAHE limits the amplification before computing the cumulative distribution function by clipping the histogram to a specific value, known as the clip limit (CDF). As a result, it is preferable to redistribute histogram sections that exceed the clip limit evenly across all histogram bins rather than discarding them. The histogram for each region is then calculated and equalized using the CDF estimate [23]. The process for equalization [21, 22] is outlined as follows.

When *P*′ and *L*′ give the pixels and grayscales count in each region, and *hi*, *j*(*l*) gives the histogram of the image (*i*, *j*) region for *l* = 1, 2, *L*1 is the histogram of the (*i*, *j*) region. The CDF scaled by (*L*1) is therefore specified for grayscale mapping as

(2) $$\begin{array}{c} F_{i,j}\left(l\right)=\frac{\left(L-1\right)}{p}\cdot \overset{l}{\underset{z=0}{\sum }}hhi,j\left(z\right). \end{array}$$

The fundamental difficulty with histogram equalization is that the area contrast is enhanced to its greatest level. (1)′s maximum slope *S*_max_ is limited to the appropriate maximum slope in order to keep the contrast at the right level. A clip limit is applied to all histograms to achieve this. The following is calculated using a clip factor (in percentages) and written as

(3) $$\begin{array}{c} \beta =\frac{p^{\prime }}{L^{\prime }}\left[1+\frac{\alpha }{100}\left(s_{\max}-1\right)\right]\text{.} \end{array}$$

Because the clip factor ranges from 0 to +100, the maximum slope in each mapping varies from ‘1' to ‘*s*_max_'. Once a histogram is received, it is spread. Its height is checked to make sure it is not too high. The CDF is then generated for grey scale mapping using the contrast's constrained histograms. The nearest region's mapping results are then mixed to map a pixel using bilinear interpolation, removing the artificially formed boundaries. It is worth noting that CLAHE's parameter settings have a significant impact on the outcome.

Figure 5 depicts the CLAHE-based enhanced image of MRI.

### 3.3. Segmentation

Individuals obtained from the previous generation through crossover, mutation, are known as survivors. We believe GA is the best contender for determining the best mix of segmentation outcomes for two reasons. The first is that differentiating between evaluation and selection conditions is difficult. GA is an optimization approach that simply requires assessing the fitness function rather than distinguishing it. This aids in the formation of innovative solutions from combinations of current results (cross-over), allowing the search to be adjusted and refocused on especially good regions once located [23].

A few critical decisions must be taken throughout any use of genetic algorithms. The genetic algorithm is carried out in four phases:

(1) Define the genotype: assessing the original population (segmentation results) and calculating each individual's fitness function (evaluation criterion).
Initial population: a group of people classified according to their genes. It is made up of the segmentation results that will be combined
Fitness function: considering its genotype, an individuals' fitness to the environment is quantified by this function.
There are several phases to the fitness computation process. Clusters are produced in the first phase based on the centres encoded in the chromosome under examination. This is accomplished by allocating each point *r*_*i*_, *i* = 1, 2,…, *n* to one of the clusters' *C*_*j*_', with ‘*Z*_*j*_' as the centre:
  (4) $$\begin{array}{c} \left|r_{i}-z_{j}\left|<\right|r_{i}-z_{p}\;|\;n=1,2\ldots K,n\neq j\text{.}\right. \end{array}$$
   Every tie is broken at random. After clustering is complete, the mean points of the various clusters replace the cluster centers stored in the chromosome. In general, the new cluster *C*_*i*_ center *G*_*i*_^*∗*^ is determined as follows:
  (5) $$\begin{array}{c} G_{i}^{*}=1\underset{ic}{\sum }\;R_{i},i=1,2,\ldots ,K\text{.} \end{array}$$
   These *G*_*i*_^*∗*^ s have now replaced the earlier *G*_*i*_ s in the chromosome. The clustering metric *M* is determined as
  (6) $$\begin{array}{c} M=\underset{xi}{\sum }\;\left\|R_{j}-G_{i}\right\|\text{.} \end{array}$$
(2) Selection of individuals. The survival of the fittest principle governs the selection of chromosomes from the mating pool in natural genetic systems. This is then transferred to the mating pool, where it will be used for subsequent genetic procedures. The proportional selection technique is used in the selection of the roulette wheel [24, 25].
(3) Mutation and crossover of individuals. Individual mutation: genes are improved in order to allow for greater environmental adaption.
  (7) $$\begin{array}{c} \prime xi+\left(\prime di{-}^{\prime }xi\right)f\left(K\right)if\;pl<0.5\text{,}\\ \prime xi-\left(\prime xi{+}^{\prime }ci\right)f\left(K\right)if\;pl>=0.5\text{.} \end{array}$$
   *p*_1_, *p*_2_: numbers present in the interval [0, 1]; *c*_*i*_, *d*_*i*_: lowest and highest limits of chromosome *x*_*i*_; *K*: the present generation; *K*_max_: the extreme number of generations; *d*: a shape parameter.
Cross-over is a probabilistic technique that produces two-child chromosomes by transferring information between two parent chromosomes.
  (8) $$\begin{array}{c} M^{\prime }=aM^{\prime }+\left(1-a\right)N^{\prime }\;N^{\prime \prime }=\left(1-a\right)M^{\prime }+aN^{\prime }\text{,} \end{array}$$
where *M* and *N* are the genotypes of the parents; *a*: a number in the range [0, 1]; *M*′, *N*′: genotypes of the parents' linear combinations.
(4) Individual/termination condition evaluation: the population's evolution can be delayed by using this criterion. Consider the stability of the population's evaluation criterion's fitness function *f* = 1/*P* offers a maximum number of iterations.  Figure 6 depicts a tumor region that was segmented using GA.

### 3.4. Feature Extraction

In this proposed method, we used the discrete wavelet transform (DWT). It is a useful tool for extracting features. The wavelet coefficient was determined from brain MR images using DWT. The wavelet locates the signal function's frequency information, which is required for classification.

#### 3.4.1. The Method Used Was the 2D Discrete Wavelet Transform

The region of interest's two-level wavelet decomposition provides four sub-bands: LL (low–low), HL (high–low), LH (low–high), and HH (high–high) (ROI). The 2D level decomposition of an image [26] provides an approximation with three detailed pictures that depict the image's low and high-level frequency components individually. These are the pictures' low-frequency components. The pictures' high-frequency components include LH1, HL1, HH1, LH2, HL2, and HH2. In the first and second layers, they provide requirements for horizontal, vertical, and diagonal directions. LL1 depicts the original picture's low-level approximation image. We repeated the procedure until we obtained the required degree of resolution.

The images were split into spatial frequency components using the 2D discrete wavelet transform. They were identified in the LL sub-bands of the spectrum. Because HL sub-bands performed better than LL sub-bands, we employed a mix of LL and HL sub-bands for enhanced analysis to characterize image-text features [27].

(9) $$\begin{array}{c} DWTp\left(s^{\prime }\right)=\left\{d\right.i,j=\sum p\left(s^{\prime }\right)h^{\prime }*i\left(s^{\prime }-2ij\right)di,j=\sum p\left(s^{\prime }\right)g^{\prime }*i\left(s^{\prime }-2ij\right)\text{.} \end{array}$$

The component property in signal *p*(*s*) corresponding to the wavelet function is represented by the coefficients *d*_*i*, *j*_. Wavelet scale and translation factors are given by the parameters *i* and *j*, respectively. The statistical features extracted are given in Table 1.

### 3.5. Feature Selection

Kennedy and Eberhart proposed an EC technique based on bio-inspired algorithms in 1995 [28]. Each bird is represented as a particle in the flock, with a swarm of particles representing a potential solution that will be optimized for a particular issue. In order to identify the global optimum, these particles are spread at random across the search space. The best personal location of the particle *g*_best_ in the swarm can identify the system's global optimum, while *P*_best_ specifies the personal best value. In each repetition, the velocity and position are updated [29, 30].

### 3.6. Classification

Biomedical images depict precise patterns of the imaged thing (for example, a brain tumor), and the object's edge is variable. Long et al. [31] proposed using skip-architecture to handle segmentation for items with precise patterns. This contributes to the development of thorough segmentation [32]. The U-Net was developed by Ronneberger et al. [32] to overcome the cell tracking problem using skip architecture as shown in Figure 7.

There are five convolutional blocks in the downsampling route. There are currently 1024 feature maps in all. With the exception of the final block, max pooling with stride 22 is done at the conclusion of each block for downsampling. Feature maps are decreased in size from 240240 to 1515. Every upsampling block begins with a deconvolutional layer of filter size 33 and stride 22. As a result, feature maps are gaining popularity. The two convolutional layers in each upsampling block lower the quantity of deconvolutional feature maps and feature maps in the encoding route. This is done in order to keep the output dimension consistent. There is no such thing as a perfectly connected layer in a network.  Table 2 lists the network's additional parameters.

## 4. Performance Analysis

Implementation of the proposed model is using hardware specifications like 11th Generation Intel® Core™ i9-11900H processor, NVIDIA® GeForce RTX 3060 and Windows 10 OS and software specifications like PyTorch and Google Collab, an open-source environment. The proposed research work uses (GA-UNET) and is compared with other models like CNN, VGG16, GoogleNet, and AlexNet under measures like accuracy, sensitivity specificity, recall, precision, *F*1-score, detection rate, TPR, FPR, and computation time, and Figure 8 is memory utilization.

Table 3 depicts the overall analysis of models for accuracy, sensitivity, and specificity shows the graphical representation of various models over the proposed method in which our method outperforms (accuracy: 0.97; sensitivity: 0.98; and specificity: 0.98).

Table 4 shows the overall analysis of various models over precision, recall, and *F*1-score.  Figure 9 illustrates the graphical representation of various models over the proposed method in which our model outperforms better (precision: 93%; recall: 86%; and *F*1-score: 93%).

Table 5 depicts the overall analysis of various models over the detection rate, TPR and FPR.  Figure 10 gives the graphical representation of various models over the proposed method in which our model outperforms (detection rate: 0.96, TPR: 0.94, FPR: 0.6).  Figure 11 depicts a graphical representation of various models over computation time and memory utilization.

## 5. Conclusion

This paper brings an effective deep learning model for brain tumor detection and classification and thereby realized the importance of advanced techniques in detection. Here, we have used the U-Net model for detecting and categorizing the brain tumor over MR multisequence image where GA is used as segmentation method that brings an effective way of detecting tumor regions, and also PSO is used in feature selection that brings better boosting to the classification stage. Experiment evaluation states our model outperforms better than other models.

## Figures and Tables

**Figure 1:** The overall architecture of the proposed system.

**Figure 2:** REMBRANDT dataset samples (a) AST, (b) GBM, and (c) OLI.

**Figure 3:** Grey scale converted image (a) and RGB image of brain tumor (b).

**Figure 4:** MRI image (a) and its skull stripped image (b).

**Figure 5:** Enhancement of image using CLAHE.

**Figure 6:** MRI image instance (a) and its segmented region using GA (b).

**Figure 7:** U-Net architecture for brain tumor classification.

**Figure 8:** Models vs. accuracy, sensitivity, and specificity.

**Figure 9:** Models vs. precision, recall, and *F*1-score.

**Figure 10:** Models vs. detection rate, TPR, and FPR.

**Figure 11:** (a) Models vs. computation time. (b) Models vs. memory utilization.

**Table 1:** Statistical features extracted using DWT.

Statistical features	Description
Mean	The sum of all pixel values in an image divided by the total number of pixels in the image [26, 27]
Standard deviations	$\sigma =\sqrt{\left(1/zn\sum_{x=0}^{z-1}\sum_{n=0}^{n-1}\left(f\left(x\right.,y\left.-\right)Z{}^{2}\right.\right)}$
Means of variance (V)	*V*_*i*_=1/*y* − 1∑_*i*=1_^*Z*^((*A*_*i*_ − *Z*)^2^)
	*V*=1/*n*∑_*i*=1_^*n*^* V*_*i*_
Inverse difference moment (IDM)	IDM=∑_*x*=0_^*m*−1^* *∑_*y*=0_^*n*−1^* *1/1+(*x* − *y*)^2^*f*(*x*, *y*)
Root mean square (RMS)	$RMS=\sqrt{\left(1/mn\sum_{x=0}^{m-1}\;\sum_{y=0}^{n-1}\;f{\left(x,y\right)}^{2}\right)}$
Smoothness	SM=1 − 1/1+(∑_*k*=0_^*m*−1^* *∑_*y*=0_^*n*−1^*f*(*x*, *y*))

**Table 2:** Parameters for U-Net.

Parameters	Value
Number of convolutional blocks	[4-5-6]
Number of deconvolutional blocks	[4-5-6]
Regularisation	[1, 1, 2, dropout]

**Table 3:** Overall analysis under accuracy, sensitivity, and specificity.

Models	Accuracy (%)	Sensitivity (%)	Specificity (%)
VGG16	82	86	92
GoogLeNet	85	90	93
AlexNet	81	89	93
CNN	92	95	97
GA-UNET (ours)	97	98	98

**Table 4:** Overall analysis under precision, recall, and *F*1-score.

Models	Precision (%)	Recall (%)	*F*1-score (%)
VGG16	84	73	87
GoogLeNet	88	76	86
AlexNet	89	79	81
CNN	90	82	88
GA-UNET (ours)	93	86	93

**Table 5:** Overall analysis under detection rate, TPR, and FPR.

Models	Detection rate (%)	TPR (%)	FPR (%)
VGG16	85	82	18
GoogLeNet	88	86	14
AlexNet	81	79	21
CNN	93	88	12
GA-UNET (ours)	96	94	6

## Data Availability

The data used in this research will be available upon request from the corresponding author.

## Abbreviations

BRATS: The Multimodal Skin Tumor Image Segmentation Benchmark
MRI: Magnetic resonance imaging
CLAHE: Contrast limited adaptive histogram equalization
GA: Genetic algorithm
TPR: True positive rate
FPR: False positive rate
PSO: Particle swarm optimization
CNN: Convolution neural network.
